# Transplantation of human umbilical cord mesenchymal stem cells to treat premature ovarian failure

**DOI:** 10.1186/s13287-021-02529-w

**Published:** 2021-08-11

**Authors:** Oldouz Shareghi-oskoue, Leili Aghebati-Maleki, Mehdi Yousefi

**Affiliations:** 1 Stem Cell Research Center, Tabriz University of Medical Science, Tabriz, Iran; 2 Student’s Research Committee, Tabriz University of Medical Sciences, Tabriz, Iran; 3 Immunology Research Center, Tabriz University of Medical Sciences, Tabriz, Iran; 4 Department of Immunology, School of Medicine, Faculty of Medicine, Tabriz University of Medical Sciences, Tabriz, Iran

**Keywords:** Premature ovarian failure (POF), Human umbilical cord mesenchymal stem cell (HUCMSC), Stem cell transplantation

## Abstract

As one of the problems and diseases for women before 40 years, premature ovarian failure (POF) could be characterized by amenorrhea, low estrogen levels, infertility, high gonadotropin levels, and lack of mature follicles. Causes of the disease involve some genetic disorders, autoimmunity diseases, and environmental factors. Various approaches have been employed to treat POF, however with limited success. Today, stem cells are used to treat POF, since they have the potential to self-repair and regenerate, and are effective in treating ovarian failure and infertility. As mesenchymal stem cell (MSC) could simultaneously activate several mechanisms, many researchers consider MSC transplantation to be the best and most effective approach in cell therapy. A good source for mesenchymal stem cells is human umbilical cord (HUCMSC). Animal models with cyclophosphamide are required for stem cell treatment and performance of HUCMSC transplantation. Stem cell therapy could indicate the levels of ovarian markers and follicle-stimulating hormone receptor. It also increases ovarian weight, plasma E2 levels, and the amount of standard follicles. Herein, the causes of POF, effective treatment strategies, and the effect of HUCMSC transplantation for the treatment of premature ovarian failure are reviewed. Many studies have been conducted in this field, and the results have shown that stem cell treatment is an effective approach to treat infertility.

## Introduction

Premature ovarian failure (POF) is one of the problems and diseases for women's reproductive health, the frequency of which has increased in recent years [1, 2]. POF is among the leading causes of female infertility prior to 40 years of age [3–5] and is characterized by amenorrhea, low estrogen levels, infertility, high gonadotropin levels, and lack of mature follicles [6–9]. These patients often have abnormal karyotypes, low levels of follicle-stimulating hormone, and decreased ovarian reserves [10, 11]. Also, negative consequences of POF include an elevated risk of cardiovascular disease, osteoporosis, and sexual dysfunction [12, 13].

Ovarian follicles include 3 types of cells: granulosa cells, oocytes, and theca cells [13]. Granulosa cells and oocytes possess FSH and LH receptors [14, 15], which are required for the growth and development of follicles [13, 16, 17].

Folliculogenesis is an organized and orderly process during which follicles grow, develop, and are prepared. Following these stages, ovulation occurs. This process changes during POF (Fig. 1) [18–21]. There are two main types of POF. In the first one, there exist few to no residual follicles, the causes of which could include genetic disorders, chemotherapy, pelvic radiation, and surgery. In the second type, there are too many follicles, and its causes include autoimmune ovarian disease, which damage maturing follicles but leaves the primordial follicles intact [13, 22, 23].

There is now evidence that some cases of this disease are due to misdiagnosis of the immune system in the ovaries [24]. Numerous evidences including endocrine disorders, histological and immunological features, transient estrogen deficiency, clinical reversibility, and manifestations of circulating ovarian antibodies in serum samples of POF-suffering women have suggested an immune source [24–27] ( Fig. 1).

## Etiology

Folliculogenesis is a regular process [28], in which primary follicles develop into secondary follicles and then into antral follicles. Next, ovulation takes place. If this natural process changes, it will lead to POF [28, 29]. POF causes are unidentified in 90% of cases; however, the number of known causes and genetic factors continue to increase (Table 1) [30].

**Table 1:** Etiology of premature ovarian failure

POF causes	Example	References
Genetic	Turner syndrome BMP15 Mutation in LH and FSH receptors Galactosemia and inhibin mutation Mutation of FOXL2, PMM2, GDF9 [31, 32]	[33–59]
Enzymatic	17α-hydroxylase, aromatase	[60]
Autoimmunity	Associated diseases: Addison’s diseases Vitiligo Myasthenia gravis Systemic lupus erythematosus Celiac disease Autoimmune polyglandular syndrome Ovarian autoantibody Zona pellucida autoantibody Immune cells imbalance: Enhancement in CD4 + T cell and B cell	[61]
Vaccination	HPV-vaccination	[62]
Chemotherapy And radiation therapy	Cyclophosphamide, Nitrogen Mustard	[63]
Environmental	Viral infections, smoking	[64, 65]

*POF* premature ovarian failure, *BMP15* bone morphogeneticprotein15, *LH* luteinizing hormone, *FSH* follicle-stimulating hormone, *FOXL2* Forkhead box L2, *PMM2* phosphomannomutase 2, *GDF9* growth/differentiation factor 9

### Genetic disorders

Few cases of family POFs have been reported, and several genetic disorders have been demonstrated in POF patients, indicating an inherited genetic disorder[31, 32]. About 20–30% of women have POF, which indicates a common hereditary POF susceptibility [33]. POF may be a heterogeneous diseases caused by mutations in a number of genes. It has been shown that with each mutation, only a few cases of POF occur [34]. Several genetic disorders, including Turner syndrome, disorder in X chromosome, fragile X syndrome, and autosomal gene mutation, have been observed in POF cases [13, 35–46].

#### X chromosome disorder

Genetically, ovarian failure is linked to X chromosomal abnormalities. These anomalies may include a small defect in chromosomal arrangement such as deletion, isochromosomes, and X-chromosome-autosomal translocation that is balanced; however, complete elimination of a X (Turner syndrome) has also been reported [47]. Complete or almost complete absence of a X chromosome in humans leads to ovarian dysgenesis, characterized by primary amenorrhea, short stature, and distinct phenotypic features [48]. In the presence of only one X chromosome, the ovarian follicles. It is declining from birth. Histological data show that ovulation in these individuals continues naturally until diplotin oocytes. It begins to combine in the follicles.

The next block in full production The follicles appear as follicular atresia [49, 50].

#### Fragile X pre-mutations

About 20% of women with fragile X pre-mutation will show symptom of fragile X-associated primary ovarian insufficiency (FXPOI) [51, 52]. Fragile X syndrome is a triple repeated disease [53]. The complete mutation results in Fragile X Syndrome, a dynamic ternary replication located in the 5% untranslated region of the FMR1 gene [54]. Premature alleles have approximately 60 to 199 replications, are unstable, and are not considered harmful in principle [37]. That is, it does not appear to be the result of a long repetition device phenotype [54]. Preliminary findings suggest that undamaged heterozygotes are at risk for premature menopause and increased twinning rates, both of which are signs of ovarian failure [54, 55]. Women with fragile X chromosome have increased FSH and decreased inhibin B levels proposing ovarian aging [56].

#### Autosomal disorder

Galactosemia is a rare autosomal recessive disease caused by a deficiency of the enzyme galactose-1-phosphate uridyltransferase (GALT).The GALT gene is located on chromosome 9p13 57. Prevalence POF in female patients with galactosemia is 70–60%. Due to the toxic effect of galactose (or one of the metabolites) on follicular structures, the initial number of oogonia decreases during fetal life, accelerating follicular atresia 58.

### Autoimmunity and POF

Some POF cases may be due to recognizing your abnormality by the immune system [59]. The evidences for an autoimmune etiology are: (1) presence of lymphocytic oophoritis [60–62]. (2) Demonstration of ovarian autoantibodies [62]. (3) Associated autoimmune disorders [62]. Oophorite is primarily characterized by cellular penetration of macrophages, natural killer cells, T lymphocytes, plasma cells, and B lymphocytes. The target of lymphocyte infestation may be class II MHC on granulosa cells. Anti-ovarian antibodies have been reported in POF [61].

Several autoimmunity diseases can cause POF [4]. It has been reported that 20% of POF patients suffer from concomitant autoimmune diseases [63], including adrenal disease, thyroid complications, and diabetes mellitus [64]. Ovarian failure might be observed as a result of autoimmune polygon syndromes type I and II. Characterization of type I syndrome is determined by adrenal insufficiency, hypothyroidism, chronic cutaneous mucosal candidiasis, hypothyroidism, and POF. On the other hand, characterization of type II syndrome is determined by thyroid autoimmune disease, adrenal insufficiency, POF, and type 1 diabetes [30, 65]. POF-related autoimmune diseases are Vitiligo, Myasthenia gravis, Addison's disease, systemic lupus erythematosus, celiac disease, and autoimmune polygon syndrome [4, 13, 62, 66–68].

### Steroidogenic enzyme defect

Defects in proteins and enzymes involved in the steroidation pathway, including 17α-hydroxylase and aromatase deficiency, could cause POF [13, 69, 70]. Steroid-producing cells (hilar cells, granulosa cells, theca internal and corpus luteum) and autoantibodies to steroid-producing cells are widely present in POF associated with Addison’s disease [71]. In autoimmune oophoritis, lymphatic infiltration is confined to secondary and antral follicles that have theca cells. This finding shows that steroid-producing cells express the antigens that stimulate the immune response [62]. Patients with enzyme deficiency other than 21-hydroxylase are very rare. In particular, a rare defect is 17,20-desmulase. Unlike other enzyme deficiencies that affect adrenal synthesis effects on corticosteroids and androgens, 17,20-desmulase inactivity affects only androgens and subsequent estrogen formation [72, 73]. Because of the activity of 17,20-desmulase and 17a-hydroxylase in the adrenal cortex, the gonads are catalyzed by a polypeptide complex. However, there are some reports of specific defects in a enzymatic activity [74]. 17,20-Desmulase deficiency syndrome is a homozygous genetic disease [75]. 17a-hydroxylase is a rare enzyme associated with puberty, primary amenorrhea, hypogonadotropism, hypertension, and hypokalemia, which could also cause ovarian failure due to defects in ovarian follicular maturation and ovarian steroid synthesis [76].

### Vaccination

Recently, POF was observed following HPV vaccination [77]. Responses of the autoimmune system to vaccines are a major aspect of autoimmune/inflammatory syndromes. HPV vaccination acts as helpers and results in POF [13, 78]. The cause is unknown in 90% of cases. Many studies have reported premature ovarian failure as a possible side effect of vaccination [79].

### Chemotherapy and radiotherapy

Among the most significant POF causes exist radiation therapy and chemotherapy used to treat cancer [80]. Although improving cancer with chemotherapy and radiotherapy in the young population leads to enhanced and durable survival [30], complications such as ovarian failure are possible. With increase in age after puberty, chemotherapy and radiation therapy could lead to POF [81]. As ovarian function is characterized by cells with rapid turnover, there is a potential similarity to tumor cells in that both are primary targets for chemotherapeutic agents. Ovarian primordial follicular cells have no ability to regenerate, and destruction of these cells leads to ovarian dysfunction which manifests as premature ovarian failure and infertility [82]. This type of treatment has several side effects, such as oocyte depletion with damage to DNA, and the disruption of functional and structural properties of oocytes [13, 81, 83, 84].

To solve this problem, in some studies to prevent premature ovarian failure due to chemotherapy (POF), temporary ovarian suppression with luteinizing hormone-releasing hormone (LHRHa) agonists has been used [85, 86].

### Environmental factors

Several environmental factors, such as viral infections, smoking, could cause infertility and POF [13, 87–90]. Studies have shown that smoking can lead to premature ovarian failure [91, 92]. Cigarette smoke comprises toxic polycyclic hydrocarbons which are harmful to germ cells and reduce follicle aging [93]. Smoking is the most widely studied toxin that alters ovarian function, and on average, the female smokers experience menopause earlier than nonsmokers suggesting a possible detrimental effect of cigarette smoking on ovarian function [91]. Among viral infections, mumps erythema could cause POF. POF was reported in 3–7% of mumps patients during an epidemic [94].

## Treatment strategies

Various treatment strategies have been performed due to the intricacy of POF disease. However, none of the treatments have been totally successful. Nonetheless, stem cell transplantation is the most effective method in this regard (Table 2) [95].

**Table 2:** Treatment strategies

Treatment strategies		References
Hormone replacement therapy	Estrogen replacement equivalents Conjugated equine estrogens	[96, 97]
	Piperazine estrone sulfate	
	Micronized 17P-estradiol	
	Transdermal estrogen path Progestin replacement equivalents	
	Medroxyprogesterone acetate	
	Duphaston Norethindrone	
	Norethisterone acetate	
	Micronized progesterone	
Melatonin therapy		[98]
(DHEA)		[99, 100]
Immunomodulation	corticosteroid for immunosuppressive	[101, 102]
	monoclonal antibodies	
	Extra-embryonic stem cells	[11, 13, 103–109]
Stem cell therapy	Induced pluripotent stem cells	
	Ovarian stem cell	
	MSC	

*DHEA* dehydroepiandrosterone, *MSC* mesenchymal stem cell

### Hormonal therapies

Application of gonadal luteinization which maintains fertility hormone-releasing hormone (LHRHa) analogs, has been suggested to reduce the incidence of POF [95, 97, 110–114]. Sex steroid deficiency with endothelial dysfunction may increase the risk of cardiovascular disease and mortality in young women and might be associated with POF. Hormone therapy restores and improves endothelial function within 6 months of treatment [115]. Estrogens play an important role in the regulation of the GH/insulin-like growth factor I (IGF-I) axis [116]. Numerous studies have shown that besides its general beneficial effects, hormone replacement therapy (HRT) increases GH secretion and precedes GH stimulation testing in postmenopausal women [117]. Estrogen replacement is suggested to treat prevent bone loss and menopausal symptoms and improve cardiovascular health in POF patients [113]. Hormone therapy increases the risk of coronary artery disease [118, 119] associated with heart disease, stroke, venous thrombosis, endometrium, breast and ovarian cancer [120–122]. In postmenopausal women, evidence of hormone-related risks in women with POF is limited. However, it is believed that the absolute risk of infection is lower in these young women and therefore the benefit/risk ratio may be higher than in older women [123].

### Melatonin

Studies have shown that melatonin increases gonadotropin levels [124], thyroid function [125], and recovery of fertility and menstruation [126]. Due to the presence of FSH, LH, androgen, and estrogen receptors on the pineal gland, it has been shown to be involved in folliculogenesis [98]. Recently, it has been shown that melatonin is produced in various tissues including reproductive tissues such as ovary and placenta [127, 128]. As the ovaries cannot produce this hormone, melatonin, which can be found in the follicular fluid, comes from blood, and the mature follicles are most probably able to accumulate it. It seems that melatonin can support ovulation [78]. Melatonin regulates the immune system both in vitro and in vivo, stimulating nonspecific humoral and cell-mediated immunity as well as antibody-mediated immunity. For this, the reason is that melatonin has been used to treat cancer [78]. The antioxidant effects and protective properties of melatonin DNA on follicles can be beneficial for female cancer survivors and prevent chemotherapy-induced fertility loss as well as premature ovarian failure [129].

### Dehydroepiandrosterone (DHEA)

As an endogenous steroid, dehydroepiandrosterone (DHEA) is derived from the zona reticularis of the ovarian monocytes and adrenal cortex in women [130]. It is very important in peripheral tissues and is produced by the conversion of cholesterol [131]. Thus, DHEA acts as a vital prohormone in ovarian follicular steroidogenesis [99]. Studies have shown that DHEA administration in patients with premature ovarian failure increases the risk of pregnancy, reduces the risk of miscarriage by reducing aneuploidy, and makes IVF treatment more successful [78, 100]. DHEA also appears to objectively improve ovarian storage. Recent animal data support androgens in enhancing pre-cleft follicle growth and reducing follicular atresia [132].

### Immunomodulation

POF treatment through immune modulation is an effective method when POF is caused by ovarian autoimmune damage [133]. Some autoantibodies that have been identified in POF are steroid-producing cell antibodies, and this antibody binds to corpus luteum, granulosa cells, hilar cells, and theca cells [111]. In this regard, monoclonal antibodies and corticosteroids are used to treat immunosuppression [101, 102, 111, 133]. Furthermore, a return of ovarian function has been observed in patients treated for myasthenia gravis using thymectomy [78]. Due to ovarian autoimmune damage, monoclonal antibodies (e.g., etanercept) are used when treating POF [78, 102, 134].

### Stem cell therapy

Due to the increased risk of cancer after using hormone replacement therapeutic and due to other side effects infertility treatments scientists have proposed other treatments, such as stem cell therapy [135, 136]. Stem cells enjoy the ability to self-repair and regenerate and are effective in treating infertility and ovarian failure [11, 137]. Recent studies on animal models of POF have shown that ovarian structure and function may improve with stem cell therapy, which could thus be an effective treatment for premature ovarian failure [138–140]. Stem cells used to treat POF include:

#### Extra-embryonic stem cells

Amniotic fluid stem cells are a multipotent population obtained from the extra-embryonic layer and proliferate faster than mesenchymal stem cells [13]. Amniotic fluid stem cell transplantation inhibits follicle atresia and maintains healthy follicles [103, 104, 141, 142].

#### Induced pluripotent stem cells

The use of human-derived ovarian granulosa cells from human-induced pluripotent stem cells could cause growth in ovarian tissue. The expression of ovarian granulosa cell markers decreases atretic follicle number and increases estradiol [11].

#### Mesenchymal stem cell

Many researchers consider mesenchymal stem cell (MSC) transplantation as the best and most successful method for cell therapy [1, 106]. Since these cells simultaneously activate several mechanisms (trophic, paracrine, immune modulation, and differentiation), they affect and improve all stages of the regeneration of damaged tissue [107]. Many researches have demonstrated that MSCs might be present throughout the body in any vascularized tissue [107]. Bone marrow-derived MSCs (BM-MSCs) are described as the "gold standard" of historically accepted MSCs [107–109]. However, there is currently active research on mesenchymal stem cells from other sources, including adipose tissue, amniotic fluid, peripheral blood and umbilical cord, tooth pulp, skin, umbilical cord tissue, synovium, placenta, endometrium, etc. [107, 143–148].

The focus of our study is on umbilical cord-derived mesenchymal stem cells (UC-MSCs), which possess an exceptional combination of prenatal and postnatal stem cell characteristics [149].

## HUCMSCs therapy

### Source

A promising source for MSCs is the human umbilical cord [150]. Unlike bone marrow stem cells, the method of collecting MSCs from human umbilical cord is faster and painless [151]. Other cells have also been reported in parts of the umbilical cord, such as vascular tissue and Wharton jelly [152, 153]. These cells have the triple activity of tissue repair, modulation of immune responses, and anti-cancer properties. HUCMCs can also be the nutrient layer of other pluripotent stem cells or embryonic stem cells [149].

Wharton umbilical cord jelly contains fibroblast-like cells and mucoid connective tissue [150]. Through the analyses of flow cytometry, it was discovered that mesenchymal cells derived from umbilical cord oxide matrix receptors (CD44, CD105) and integrin markers (CD29, CD51) are not hematopoietic markers (CD34, CD45) [150].

**Fig. 1:** Folliculogenesis: ovarian follicles enjoy an immature oocyte and somatic cells. Ovarian follicle maturation illustrates the passage of several small primordial follicles into pre-ovulatory follicle, which ultimately results in the maturation of oocyte

### The importance of UCMSC

Human mesenchymal stem cells (MSCs) have recently received a great deal of attention due to their enormous therapeutic potential. Less ethical issues, painless obtaining of the abandoned umbilical cord, and lack of immunity are prominent benefits of hUCMSC compared to other MSC resources [154]. The ability to modulate immune responses makes hUCMSC an important stem cell resource for allogeneic transplantation without immunosuppression [155]. There is no evidence of an immunological response and no evidence of increased dose and frequency of hUCMSCs used in patients [156]. Based on the evidence gathered, stem cells improve ovarian function due to their paracrine effects rather than differentiating into specific cells [157]. Studies on stem cell-derived secretory agents report that the secretion of microscopes and exosomes is present in the stem cell culture medium known as the conditioned medium (CM) [158]. The contents of these vesicles secreted by mesenchymal stem cells (MSCs) include cytokines and growth factors, signaling lipids, messenger RNAs (mRNAs), and regulatory miRNAs [159]. These factors are involved in cell–cell communication, cellular signaling, and changes in cell or tissue metabolism. CM can enhance tissue/limb repair under different conditions [160]. CM has several advantages over stem cells. CM eliminates stem cell side effects on tumor cells, such as differentiation into other stromal cells, enhances the metastatic capabilities of tumor cells, and stimulates epithelial–mesenchymal transmission of tumor cells [161, 162]. hUCMSC-CM can regulate G-CSF expression in granulosa cells and reduce granulosa cell apoptosis [163]. The anti-apoptotic effects of G-CSF have been reported in vascular endothelial cells, heart and nerve cells [164]. The PI3K/Akt pathway is activated in granulosa cells, thereby reducing granulosa cell apoptosis [165]. In addition, hUCMSCs have multifunctional stem cell characteristics that can be differentiated into several breeds under different conditions of differentiation [166, 167]. Some studies have also shown that hUCMSCs differentiate into oocyte-like structures and express germ cell-specific mRNA and protein markers. hUCMSC increases the proliferation of damaged human endometrial stromal cells (ESCs) and significantly reduces the percentage of apoptosis when cultured with them [168]. hUCMSC may restore endometrial damage through secretion of vascular endothelial growth factor (VEGF) and anti-apoptosis [169]. In one study, POF model rats were injected with different concentrations of UCMSC. Follicular morphology, ovarian function, hormonal secretion, and proliferation and apoptosis of granulosa cells were assessed. It was demonstrated that follicular growth was considerably enhanced after UCMSC transplantation and rat estrous cycle returned to normal. Moreover, the levels of progesterone (P4), estradiol (E2), and antimalarial hormone (AMH) were significantly increased [170,  171] in the serum. UCMSC transplantation also reduces granulosa cell apoptosis and granulosa cell proliferation [22]. These results further confirm the increase in tissue regeneration and cellular growth factors and present theoretical foundations for applying stem cells clinically to treat POF [171–174]. HUCMSC transplantation can also restore chemotherapy-damaged ovaries. Improved ovarian function in the rat model of premature ovarian failure (POF) is largely due to cytokines produced by hUCMSCs through the paracrine mechanism rather than direct differentiation into germ cells [175]. In the process of transplantation, endometrial acceptance refers to the ability of the endometrium to allow embryos to implant during a particular period [176, 177]. Embryo implantation is similar to allograft transplantation, which is also a complex process involving many immune system regulating factors such as Th1/Th2 cytokine imbalances. Natural uterine killer cells (uNK) play an important role in maintaining the Th1/Th2 cytokine balance in the local endometrial immune response. uNK cells are a group of specific cells in the endometrial stroma where most uNK cell phenotypes are stained as CD56 + CD16 − [ 178–180]. uNK cells proliferate rapidly in the secretory stage and early pregnancy. If uNK cells are activated by certain pathological factors, the cells secrete cytotoxic factors to lead to an imbalance of Th1/Th2 cytokines. Consequently, this reduces the effect of Th1 cytokines on endometrial receptivity and embryo implantation failure [180, 181]. As reported, changes in endometrial acceptance depend on the specific spatial and temporal expression of certain gene sets in the endometrium. Among them, the HOXA10 gene is used as a molecular marker to measure endometrial receptivity [182]. Some studies have shown that large numbers of immune cells invade ovarian tissue in mice with premature insufficiency, including T lymphocytes [183, 184], B lymphocytes, and normal killer cells [25]. It has also been reported that the balance of Th1/Th2 cytokine expression in the T lymphocyte subtype is abnormal in patients with POF [185]. Studies have shown that immune regulation in Th1/Th2 cytokine balance and uNK cell expression is involved in improving ovarian function and improving endometrial receptivity after hUCMSC transplantation in POF mice [186]. In 2019, Yang Lei et al. used a collagen scaffold filled with hUCMSCs (collagen/hUCMSC) in ovulating POF mice (six-week-old female C57BL/6 mice), which maintained ovarian function, and enhanced anti-Mullerian hormone (AMH) and estrogen (E2) levels. It also increased the volume of ovaries and the amount of antral follicles. Immunohistochemical assessment showed that collagen/h-UC-MSC transplantation promoted granulosa cell proliferation, which is crucial for follicle maturation [171]. In 2020, Wang Wei et al. used different concentrations of UCMSC in POF rats (female rats). It was shown that the estrous cycle of rats was restored to natural, and follicular growth was considerably enhanced following UCMSC transplantation. Moreover, the levels of progesterone (P4), 17-estradiol (E2), and anti-molar hormone (AMH) were considerably increased in the serum. UCMSC transplantation, likewise, reduced granulosa cell apoptosis and proliferation [172]. In 2020, Shen and Dai Cao used HUCMSCs in POF mice (female BALB/c mice) with the aim of repairing ovarian injury following chemotherapy. It has been demonstrated by several experiments that umbilical cord-transplanted stem cells are capable of proliferating and migrating into the ovaries, improving ovarian function, increasing the amount of follicles and granulosa cells on all ovary levels, and improving endocrine function [173]. In 2020, Yin Wu et al. used UCMSCs to restore the ovarian function in POF mice (C57BL/6). Transplantation increases the number of functional follicles and the regular production of hormones [187]. In 2019, Zheng Fu et al. used UCMSC transplantation after chemotherapy-induced ovarian damage. The study showed that UCMSC transplantation improves folliculogenesis and disturbed secretion of hormones in POF mice (C57BL/6) [106]. In 2019, Yang Du et al. used HUCMSC-MVs to restore ovarian function in a female mouse model with chemotherapy-induced POI. The results showed that HUCMSC-MV transplantation can increase weight of the body, enhance the amount of ovarian follicles (early follicles, growing and ovulating before ovulation), stimulate ovarian angiogenesis, and restore the unstable estrous cycle of POI mice [188]. In 2019, Jalalie Rezaie et al. used human umbilical cord vein MSCs (HUCV-MSCs) in several parts of the ovarian tissue in mice (adult female C57BL/6 mice) who had cyclophosphamide (CTX)-induced POF. The results showed that MSCs were capable of migrating to injured tissues and repairing them through the modulation of immune system and secretion of growth factors [189]. In 2016, Elfayomy Almasry et al. used the human umbilical cord blood (HCB) MSCs to evaluate their effect on ovarian epithelium following paclitaxel-induced ovarian failure in POF rats. The results showed that HCB-MSCs were capable of restoring ovarian function following paclitaxel injection [190]. In 2013, Wang Yu et al. used UCMSC to treat POF rat models and the results

## Methods

To model POF mice, random division of the female BALB/c mice into two groups was performed: the control group and the POF group. POF mice were injected with CTX intraperitoneum. The control group was injected with normal saline instead of CTX, without there being any treatment or negative control [149, 192]. Infant cord tissue was taken with the consent of the donor. Manual dissection of the umbilical cord into small parts was performed. Tissues fragments were cultured in low glucose Dulbecco’s modified Eagle’s medium and with fetal bovine serum penicillin, combined with streptomycin. After obtaining HUCMSC colonies, flow cytometry was used for the analysis of UC-MSC level markers. Cells with (PE) and (FITC) against human CD13,CD34,CD45, CD73, CD90, CD105, CD146, and HLADR were incubated [190]. Scaffolds (collagen type 1) were prepared from the molecule laboratory [171, 193]. Collagen/UC-MSC transplantation was performed for mice [2, 171, 175, 190]. Following transplantation, rat hormone levels and number of ovarian follicles were measured, and ovarian morphology was assessed by hematoxylin and eosin (HE) staining (Fig. 2) [175].

**Fig. 2:** The use of stem cell therapy to treat POF. The application of stem cells for the treatment of POF mice and renewing follicles after stem cell transplantation. Stem cell therapy results in the treatment of POF mice

## Conclusion

POF hugely affects mental and physical health of young women. Women with this condition usually use hormone therapy to reduce the symptoms of estrogen deficiency, which is not very effective. Therefore, we must look for better alternatives to treat the disease. Many studies have been performed in this field, the results of which propose stem cell therapy as more effective compared to other methods. Since these cells have the potential for self-improvement and regeneration and can improve ovarian function, increase the number of follicles, increase sex hormone levels, and reduce granulosa cell apoptosis, they could be employed to treat POF and infertility. In most studies, mesenchymal stem cells are used due to the facile access to these cells and their differentiation in most tissues. Our study was focused on mesenchymal cells derived from the human umbilical cord. Researchers have achieved decent results in this field, and thus, it is hoped that researchers can find a definite cure for this disease.

## Data Availability

Data sharing is not applicable to this article as no new data were created or analyzed in this study.

## Abbreviations

AMH: Anti-Müllerian hormone
BM-MSCs: Bone marrow mesenchymal stem cells
CTX: Cyclophosphamide
DHEA: Dehydroepiandrosterone
E2: Estradiol
FITC: Fluorescein isothiocyanate
FSH: Follicle-stimulating hormone
HCB: Hexachlorobenzene
HE: Hematoxylin and eosin
HPV: Human papillomavirus infection
HUCMSC: Human umbilical cord mesenchymal stem cells
HUCMSC-MVs: Human umbilical cord mesenchymal stem cell-derived microvesicles
LH: Luteinizing hormone
LHRHa: Luteinizing hormone-releasing hormone analog
Name: Mesenchymal stem cell;
P4: Progesterone
PE: Phycoerythrin
POF: Premature ovarian failure
POI: Premature ovarian insufficiency
UC-MSCs: Umbilical cord mesenchymal stem cells
VEGF: Vascular endothelial growth factor
